# A Study on the Effects of a Cartoon Text Version of Health Education Manual with Sandplay on the Psychological Status and Cognitive Function of Children with Attention Deficit Hyperactivity Disorder

**DOI:** 10.1155/2022/1816391

**Published:** 2022-09-12

**Authors:** Lei He, Lifeng Huang

**Affiliations:** Guangzhou Women and Children's Medical Center Pediatric Clinic, Guangzhou 510000, Guangdong, China

## Abstract

**Purpose:**

The study aimed to examine the effects of a cartoon text version of a health education manual with sandplay on the psychological status and cognitive function of children with attention deficit hyperactivity disorder (ADHD).

**Methods:**

Eighty cases of children with ADHD admitted from February 2019 to September 2021 were selected for the study. They were numbered according to the order of consultation, and after obtaining family consent, they were divided into the control group (*n* = 40) and the observation group (*n* = 40) using the random number table method. The control group received only medication and verbal health education, while the observation group received a cartoon text version of the health education manual together with sandplay on top of the above, and both groups were treated for 30 weeks. The attention test results and the Swanson, Nolan, and Pelham-IV rating scales (SNAP-IV) were used to assess the effectiveness of the treatment for both groups of children. The awareness rate of health education knowledge of children and their families in both groups was counted. The Conners Parent Symptom Questionnaire (PSQ) and the Combined Raven's test (CRT) were used to assess the psychological status and cognitive functioning of the children in both groups.

**Results:**

After treatment, the response time, the number of errors, and the number of missed alarms in the attention test results were lower in the observation group than in the control group (*P* < 0.05). After treatment, the inattention, antagonism and defiance, and impulsiveness and hyperactivity scores on SNAP-IV were lower in the observation group than in the control group (*P* < 0.05). After treatment, the knowledge of disease and treatment, medical and nursing cooperation, safety and protection, and dietary precautions were higher in the observation group than in the control group (*P* < 0.05). After treatment, the learning problems, conduct problems, psychosomatic problems, anxiety, impulsivity-hyperactivity, and hyperactivity index scores on the PSQ were lower in the observation group than in the control group (*P* < 0.05). After treatment, the A, B, C, D, and E theme scores in the CRT were higher in the observation group than in the control group, and the IQ score was also higher in the observation group than in the control group (*P* < 0.05).

**Conclusion:**

The cartoon text version of the health education manual with sandplay can significantly improve the attention deficit, hyperactive behaviour, psychological status, and cognitive function of children with ADHD on the basis of pharmacological treatment, which has a good clinical application.

## 1. Introduction

Attention deficit hyperactivity disorder (ADHD) is one of the most common neuropsychiatric disorders in children. The main manifestations are that attention that is not commensurate with age is easy to be distracted, the attention span is reduced, excessive activities, emotional impulses, and willfulness. Children are often accompanied by different degrees of psychological behaviour abnormalities, cognitive dysfunction, and learning difficulties, and their intelligence is normal or close to normal [1, 2]. At present, most children and their families do not have a good understanding of ADHD. They still believe that the clinical symptoms of the children are poor ideological and moral character and do not accept discipline. Parents and teachers often give rude education. Students, relatives, and friends are more likely to alienate and discriminate against them. Children cannot correctly face their diseases, which will continue to affect their mental health, behaviour, and cognitive function. It seriously affects the quality of life and normal development of children.

At present, there are many methods to treat ADHD. In addition to drug treatment, there are multiple targeted treatment methods [3]. Sandplay is a form of therapy that is fun and educational and has become a widely accepted form of therapy as the concept of humanistic therapy continues to develop [4, 5]. In addition, the young age and poor self-management skills of children with ADHD, as well as the mobility of their family chaperones, often due to time constraints, make it difficult for many children with ADHD to receive verbal health education and behaviour management guidance. In recent years, the department has been actively using the cartoon text version of the health education manual to treat 40 cases of children with ADHD together with sandplay, which has not only enabled all children and their accompanying family members to learn the relevant health education and care knowledge and reduce the safety risks but also effectively improved the clinical treatment results of the children, as reported below.

## 2. Materials and Methods

### 2.1. General Materials

Eighty cases of children with ADHD admitted from February 2019 to September 2021 were selected for the study. Inclusion criteria were as follows: ① those who met the Diagnostic and Statistical Manual of Mental Disorders, 5th edition (DSM-5) [6] criteria for the diagnosis and staging of ADHD in the United States; ② those with an intelligence quotient (IQ) score of 85 to 110 on the Wechsler Intelligence Scale for Children (WISC-CR) [7]; ③ ages 6 to 12 years; ④ those who accepted the treatment with good compliance and completed the assessment. Exclusion criteria were as follows: ① exclusion of children with mental retardation, epilepsy, organic encephalopathy, autism, affective disorders, schizophrenia, tic disorders, digestive disorders, and malnutrition; ② children with a history of psychotropic substance use; ③ those who had received other medication before the study. All children were numbered according to the order of consultation, and after obtaining family consent, they were divided into the control group (*n* = 40) and the observation group (*n* = 40) by using the random number table method. The comparison of general information between the two groups is shown in Table 1, and none of them were significantly different and comparable (*P* > 0.05).

### 2.2. Methods

1. The control group received only medication and verbal health education. The drug of choice was methylphenidate hydrochloride extended-release tablets (Janssen-Cilag Limited, State Drug Administration J20120028), administered orally at a starting dose of 18 mg/d once a day in the morning for 30 weeks, and during that time, the child's clinical response and drug tolerance were strictly monitored and the dose was adjusted as necessary. Oral education of health education knowledge: according to the requirements of routine nursing, the children and their families were provided with health education through oral explanation, public class lectures, and action demonstrations.
2. The observation group received a cartoon text version of the health education manual together with sandplay on top of the above. Cartoon text version of the health education manual: the main contents of health education (e.g., greetings on admission, names, and contact details of the attending physician and responsible nurse, information on the child's illness and treatment, knowledge on the cooperation between health care and nursing, safety and protection, and dietary precautions) were made into the cartoon text version of the health education manual, and the cartoon text version of situation maps in different situations with cartoon characters (e.g., GG Bond, Pleasant Goat, Bear senior, and Bear junior) loved by children was drawn. Sandplay: the therapists were counselors with practical experience in sandplay psychotherapy. The sandplay room was configured according to international standards, with toy shelves on both sides containing household items, transport, military machinery, and plant and animal toys, creating a very safe, free, and relaxing environment for children to draw on sandplay. Once the child entered the sandplay room, the therapist instructed him/her on the basic operation of the sand play and guided him/her to focus on the game, asking him/her to signal when he/she had finished playing, while the nursing staff took notes, and the parents observed and did not disturb the child's play. The length of the game was controlled at ≤60 min/time. After the game, the nursing staff asked the child what he or she had shaped and induced him or her to describe his or her feelings during sandplay therapy so that the nursing staff could understand his or her personality and signs and purposefully set different sandplay themes each week to stimulate the child's imagination and creativity, 1 time/week for 30 weeks of treatment.

### 2.3. Assessment Indicators

1. Attention test results: the integrated visual and auditory continuous performance test (IVA-CPT) [8] was administered to all children after treatment for 12 minutes to measure visual, auditory, and sustained attention. The response time, the number of errors, and the number of missed alarms were automatically recorded by the program.
2. ADHD rating scale 4th edition (Swanson, Nolan, and Pelham-IV rating scales, SNAP-IV) scores: the SNAP-IV rating scales [9] had 26 items including 3 areas of inattention, antagonism and defiance, and impulsiveness and hyperactivity. Each entry was rated from 0 to 3 according to the frequency of occurrence, with higher scores indicating more severe ADHD in individuals.
3. Awareness rate of health knowledge: after treatment, the awareness of the children and their families of the knowledge of disease and treatment, medical and nursing cooperation, safety and protection, and dietary precautions were counted in both groups.
4. Conners Parent Symptom Questionnaire (PSQ) scores: PSQ [10] had 48 entries including six factors learning problems, conduct problems, psychosomatic problems, anxiety, impulsivity-hyperactivity, and hyperactivity index. Each entry was scored from 0 to 3, with higher scores indicating more serious problems in this area in children. The scale had been extensively tested for clinical validity and was adequate for general assessment. The PSQ was used in this study to assess the behavioural problems and psychological status of children with ADHD.
5. Combined Raven's test (CRT): the main tests were divided into five groups of themes: A (perceptual discrimination, graphical comparison, and graphical imagination), B (similarity, comparison, and graphical combination), C (comparison, inference, and graphical combination), D (series relations, graphical sets, and sums), and E (abstract thinking skills). Each group consisted of 12 questions and the test lasted 30 to 40 minutes, with 1 mark for a correct answer and 0 marks for an incorrect answer. The scores were added to get the original score. The original total score of the child was converted into the percentage grade according to the percentage grade norm table, and then, the percentage grade was converted into the corresponding IQ value according to the IQ norm table. CRT was used in this study to evaluate the cognitive function of children with ADHD.

### 2.4. Statistical Methods

The data analysis software was SPSS 22.0, and the plotting software was GraphPad Prism 8.0. Statistical information was described in (%) and adopted the *χ*^2^ test, and measurement information was expressed in (*x* *±* *s*) and adopted the *t*-test. A two-sided test of *P* < 0.05 was considered a statistically significant difference.

## 3. Results

### 3.1. Comparison of Attention Test Results between the Two Groups

After treatment, the response time, the number of errors, and the number of missed alarms in the attention test results were lower in the observation group than in the control group (*P* < 0.05) (Figure 1).

### 3.2. Comparison of SNAP-IV Scores between the Two Groups

After treatment, the inattention, antagonism and defiance, and impulsiveness and hyperactivity scores on SNAP-IV were lower in the observation group than in the control group (*P* < 0.05) (Figure 2).

### 3.3. Comparison of the Awareness Rate of Health Education Knowledge between the Two Groups

After treatment, the knowledge of disease and treatment, medical and nursing cooperation, safety and protection, and dietary precautions were higher in the observation group than in the control group (*P* < 0.05) (Figure 3).

### 3.4. Comparison of PSQ Scores between the Two Groups

After treatment, the learning problems, conduct problems, psychosomatic problems, anxiety, impulsivity-hyperactivity, and hyperactivity index scores on the PSQ were lower in the observation group than in the control group (*P* < 0.05) (Figure 4).

### 3.5. Comparison of CRT Scores and IQ Values between the Two Groups

After treatment, the A, B, C, D, and E theme scores in the CRT were higher in the observation group than in the control group, and the IQ score was also higher in the observation group than in the control group (*P* < 0.05) (Figures 5 and 6).

## 4. Discussion

ADHD, also known as hyperactivity disorder, is the result of a combination of genetic, biological, psychological, social, and environmental factors that contribute to the disease. The disease is characterized mainly by hyperactivity during school age, more pronounced attention deficit during primary school, and impulsivity, impatience, restlessness, and attention deficit in adulthood, which can lead to poor academic performance, poor peer relationships, and social exclusion, and then conduct disorder and antisocial personality disorder and seriously affect children's physical and mental health, as well as work and learning in adulthood [11].

The nonpharmacological treatment of ADHD with few side effects and the little economic burden has now attracted much attention from the parents of low-age children and scholars at home and abroad. In 2001, the American Academy of Pediatrics [12] recommended behavioural interventions for preschoolers (4 to 5 years old); for primary schools children (6 to 11 years old) using FDA-approved medications for ADHD and/or behavioural interventions by parents and/or teachers, with a combination of both resulting in better outcomes. Our latest guidelines for the prevention and treatment of ADHD also place special emphasis on the use of behavioural interventions for children up to the age of 12 years [13]. The results of this study showed that after treatment, the response time, the number of errors, and the number of missed alarms in the attention test results were lower in the observation group than in the control group, and the scores of inattention, antagonism and defiance, and impulsiveness and hyperactivity on SNAP-IV were lower in the observation group than in the control group. This suggests that medication combined with a psychological-behavioural intervention of the cartoon text-based health education manual and sandplay can improve the child's ADHD symptoms better than medication alone.

Health education aims to improve patients' compliance with treatment, reduce the psychological burden, and enhance treatment outcomes [14]. However, in our clinical practice, most of the guardians of children are shared by grandparents and parents, with grandparents' cognitive and information-receiving abilities being relatively poor and the parents spending relatively little time with them, thus making health education less effective. In recent years, our department has printed content requiring health education and behavioural guidance in simple, heartwarming language on a cartoon background booklet that children like. This attracts the child's attention and can promote active access to health education knowledge by the child and his or her chaperones, enabling health education guidance to be put into practice and increasing the rate of knowledge of health education.

Sandplay is a bridge for adults to connect children's inner world before children's expressive language functions are fully mature [15]. In sandplay, a quiet treatment environment and a self-pleasant play course allowed all children to feel their dominant strength and thus gain a sense of controllability, which improved gradually as a “ sense of controllability ” was recovered. Sandplay provides a way for children to vent bad feelings and express aggressive behaviour, allowing them to channel their excess energy into appropriate behaviour and reduce hyperactivity, impulsivity, and aggressive behaviour. During the production of sandplay, those that are attractive, palpable, and mobile offer the ability to stimulate children's brain nerves with tactile and muscular motion senses to enhance attention. In addition, sandplay can also develop children's imagination and creativity, as well as help with logical thinking and language skills.

The PSQ is an assessment tool used to screen children for behavioural problems (especially ADHD) [16]. This study applies it to the assessment of behavioural problems and the psychological status of children with ADHD. The CRT is a test instrument with special features not found in general text-based intelligence tests. It can be used in situations where verbal communication is difficult and is suitable for a variety of cross-cultural comparative studies, or for testing the cognitive functioning of certain special populations, and is suitable for ages 5 to 75 years [17]. This study uses CRT for the assessment of cognitive function in children with ADHD. The results showed that after treatment, the observation group had better scores for each factor item in the PSQ, CRT, and IQ values than the control group. This suggests that the cartoon text version of the health education booklet combined with sandplay therapy, in addition to medication, can significantly improve the psychological status and cognitive function of children with ADHD, as well as improve their intelligence.

Sandplay therapy has the following advantages: ① the games are fun and rich, in line with the psychological characteristics of the age group of the child, who rarely perceives them as therapy and participates in them as a game, ensuring that the therapy is quiet, comfortable, relaxing and enjoyable, and therefore highly acceptable and cooperative [18]. ② The therapist's company can fully induce the child to create works that vividly reflect the child's inner world. Through the construction of a safe, warm, supportive, custodial, empathic, and caring space, the child removes the psychological barrier and fully shows his or her inner self, and the negative personality and character behaviour are fully eased [19]. ③ Objective information reference: in conventional therapy, the child has a psychological barrier, and it is difficult for the practitioner to read the child's inner world from just a few words while using the work as an objective information reference; through the work, the therapist can clearly observe the child's inner world. Then, according to the cognitive-behavioural theory of psychology, the therapist provides targeted guidance to help the child find strength in self-growth and promote deep personality integration, which helps the child's emotional and mental stability and behavioural and cognitive improvement after treatment [20].

## 5. Conclusion

The cartoon text version of the health education manual with sandplay can significantly improve the attention deficit, hyperactive behaviour, psychological status, and cognitive function of children with ADHD on the basis of pharmacological treatment, which has good clinical application.

## Figures and Tables

**Figure 1:** Comparison of attention test results between the two groups. *Note*. The symbol ^*∗*^indicates a statistically significant difference between the two groups.

**Figure 2:** Comparison of SNAP-IV scores between the two groups. *Note*. The symbol ^*∗*^indicates a statistically significant difference between the two groups.

**Figure 3:** Comparison of the awareness rate of health education knowledge between the two groups. *Note*. The symbol ^*∗*^indicates a statistically significant difference between the two groups.

**Figure 4:** Comparison of PSQ scores between the two groups. *Note*. The symbol ^*∗*^indicates a statistically significant difference between the two groups.

**Figure 5:** Comparison of CRT scores between the two groups. *Note*. The symbol ^*∗*^indicates a statistically significant difference between the two groups.

**Figure 6:** Comparison of IQ values between the two groups. *Note*. The symbol ^*∗*^indicates a statistically significant difference between the two groups.

**Table 1:** Comparison of general information between the two groups.

Items	Control group (*n* = 40)	Observation group (*n* = 40)	*t*/*χ*^2^	*P*
Age (years old)	9.30 ± 1.73	9.23 ± 1.27	0.206	0.837
Disease duration (months)	14.38 ± 4.16	14.60 ± 3.75	0.248	0.805
Male (*n*, %)	24 (60.00)	26 (65.00)	0.213	0.644
Type (*n*, %)			1.461	0.482

Attention deficit type	24 (60.00)	23 (57.50)		
Hyperactive-impulsive type	2 (5.00)	5 (12.50)		
Combination type	14 (35.00)	12 (30.00)		

## Data Availability

The data supporting this study are available to the corresponding author on reasonable request.
